The article "The Application Value of Contrast-Enhanced Ultrasound in Testicular Occupied Lesions" was published in 2021. Journal: Comput Math Methods Med.

# The Application Value of Contrast-Enhanced Ultrasound in Testicular Occupied Lesions

**DOI:** 10.1155/2021/9962970

**Published:** 2021-06-11

**Authors:** Qiping Liu, Huiling Gong, Hui Zhu, Chunyan Yuan, Bin Hu

**Affiliations:** ^1^Department of Ultrasound, Minhang Hospital, Fudan University, Shanghai 201199, China; ^2^Department of Pathology, Minhang Hospital, Fudan University, 170 Xin-Song Road, Shanghai 201199, China

## Abstract

**Objective:**

To discuss the clinical application value of contrast-enhanced ultrasound (CEUS) in testicular occupied lesions.

**Methods:**

Nine conventional-ultrasound-found testicular occupied lesions which underwent CEUS meantime were analyzed retrospectively. The CEUS perfusion pattern was compared with the surgical pathological result or follow-up findings.

**Results:**

Among all the 9 testicular occupied lesions, there were 5 testicular malignant tumors, 1 testicular benign tumor, 1 testicular tuberculosis, and 2 testicular hematomas. CEUS diagnosed 6 testicular malignant tumors, 1 testicular benign tumor, and 2 testicular hematomas, and its diagnostic accuracy was about 88.9%.

**Conclusion:**

CEUS has high clinical application value in the differential diagnoses of benign and malignant testicular occupied lesions.

## 1. Introduction

Testicular tumors are relatively rare, typically speaking, which accounts for only 1% of all sorts of malignant tumors of the whole body, but they are the most common solid tumors in young men aging from 20 to 40 years old, almost all of which are malignant [1]. The benign and malignant diseases formed by testicular cysts need to be distinguished by differential diagnosis and etiology [2]. The benign diseases of testicular cystic space-occupying lesions are testicular reticular dilatation, cystic dysplasia, epidermoid cysts, simple solid intratesticular cysts, and albuginea cysts [3]. In most benign testicular lesion diagnosis cases, it is recommended to use an organ-conserving surgical therapy or an observational watch-and-wait strategy [4].

Due to its convenience and noninvasive advantages, ultrasound examination has been widely used in the diagnosis of testicular occupied lesions, and it has become an important method of distinguishing benign and malignant testicular tumors. Contrast-enhanced ultrasound (CEUS) is a safe, relatively cheap, and widely available imaging technology [5]. It uses a dedicated imaging ultrasound sequence and FDA-approved contrast agent microbubbles [6]. It can detect and characterize malignant focal liver lesions and has a high diagnosis [7]. The current evidence shows that CEUS can accurately distinguish solid and cystic kidney masses [8], and CEUS is very suitable for proving the tumor microvessels associated with malignant kidney masses [9]. CEUS studies the blood flow of the prostate, visualizes prostate cancer, and performs targeted biopsy and has shown its diagnostic value for prostate cancer [10]. Various changes in CEUS (such as DCE-US and ultrasound molecular imaging) are emerging for quantitative monitoring of treatment effects and possible early detection of cancer [11–13]. CEUS can dynamically display the tiny blood circulation inside tumors [14], which benefits identifying the nature of the tumor. In this article, we retrospectively analyzed 9 cases of testicular occupied lesions confirmed by surgery or follow-up in recent years in our hospital. By CEUS, we detected the blood flow of testicular occupied lesions, observed their perfusion patterns in order to explore the clinical application value of CEUS in testicular occupied lesions.

## 2. Materials and Methods

### 2.1. Patient Population

Collecting testicular occupied lesion cases during November 2013 and September 2020, which were detected by routine ultrasound examination in our hospital, we had 9 patients in all. Five cases had lesions in the right testicles and 4 cases in the left ones. Besides these, 2 cases had a history of testicular trauma. Patients were aged from 30 to 59 years old, 38 years old on average. The size of lesions was 52 mm × 25 mm × 25 mm maximum and 8 mm × 3 mm × 7 mm minimum. CEUS was performed in all 9 cases.

### 2.2. Imaging Techniques

Aplio 500 (Toshiba, Japan) ultrasonic scanner with a 5~14 MHz linear transducer was used for an ultrasound examination. It was also equipped with color Doppler flow imaging (CDFI) and CEUS imaging software. The patients lay supine on the couch, fully exposing the scrotums. We scanned the scrotums from multiple sections and angles. First, the testicular scan was performed with conventional ultrasound, focusing on the observation of the location, size, number, morphology, boundary, and internal echo of the lesions. CDFI was then used to observe the distribution of blood flow in and around the lesions. After that, we switched it to CEUS mode. SonoVue was used as the contrast agent. 5 ml of normal saline (NS) was injected before use, and 2.4-3.0 ml of the mixture was extracted after shaking. After windowing the best image of the lesion, the extracted mixture was injected rapidly through the cubital vein, followed by 5 ml of NS, and a timer was set simultaneously. After contrast agent injection, real-time images were observed continuously for 3-5 mins. All images were archived for offline analysis. Two to three experienced senior sonographers repeatedly reviewed the playback clips, so as to dynamically observe the changing trend of contrast agent; summarized the perfusion pattern of contrast agent in terms of time and echo intensity; and analyzed the CEUS results. Finally, the medical history and pathological data were followed up for comparative analysis.

### 2.3. Imaging Interpretation

CEUS descriptions: (1) the enhancement intensity of the mass was divided into hyperenhancement, isoenhancement, hypoenhancement, and no enhancement; (2) the homogeneity of enhancement was divided into homogeneous enhancement and heterogeneous enhancement; (3) compared with normal testicular tissues, the entering time and washout time of the contrast agent were observed, and the enhancement phase of mass was divided into fast-in and fast-out, fast-in and slow-out, slow-in and fast-out, slow-in and slow-out, etc.

## 3. Results

### 3.1. Manifestation of CEUS

Testicular occupied lesions showed hypoechoic or heterogeneous echogenic regions in the testis on gray scale ultrasonography and weak or rich blood flow signals in some cases on CDFI (Figure 1). There were 5 cases of malignant testicular tumor, among which 4 cases presented fast-in and fast-out enhancement on CEUS, and 1 case presented fast-in and slow-out enhancement and heterogeneous hyperenhancement at the peak time (Figure 2). All these 5 cases were indicated to be malignant testicular tumors through CEUS. There was 1 benign testicular tumor case that presented fast-in and fast-out enhancement on CEUS and slightly heterogeneous hyperenhancement at the peak time. It was indicated to be a benign lesion by CEUS. There was 1 testicular tuberculosis case on which CEUS showed fast-in and fast-out enhancement and heterogeneous hyperenhancement at the peak time. It suggested a malignant testicular tumor. There were 2 testicular hematoma cases on which no enhancement was seen during the entire process (Figure 3). Combined with the medical history, they were thought to be testicular hematoma cases.

### 3.2. Diagnostic Accordance Rate

All 9 patients with testicular occupied lesions were followed up or surgically treated.

Six cases were suggested as malignant tumors by CEUS, and 5 of them were confirmed correct by surgical pathology (including 3 seminoma cases and 2 mixed germ cell tumor cases). The other one was testicular tuberculosis confirmed surgically. CEUS showed a benign tumor, and the surgical pathology was an adenomatoid tumor of the testis. Two cases of testicular hematoma were confirmed by follow-up observation. The CEUS diagnostic accordance rate of testicular occupied lesions was approximately 88.9% (8/9).

## 4. Discussion

Testicular tumors are classified into germ cell and nongerm cell types. Germ cell testicular tumors account for the majority of them, of which about 95% are malignant, and seminoma is the most common type [15]. Nongerm cell tumors are so rare, accounting for only 3.5%, that they contain fibroma and hemangioma, etc. [16]. The testicular malignant tumor has no active biological behavior that it is prone to have hematogenous and lymphatic metastases. Once it metastasizes, the prognosis is poor.

Early detection, diagnosis, and treatment are the keys to improve the cure rate of testicular tumors [17]. Ultrasonic diagnosis has a high accordance rate and has become the preferred method for the diagnosis of testicular tumor [18]. Conventional gray scale ultrasound can measure the size of the testicular mass and observe its echo, boundary, shape, etc. CDFI can show the blood supply inside the tumor. CDFI could show 1-2 mm blood vessels at most, but the effort in showing smaller blood vessels was for naught [19]. SonoVue, a new ultrasound contrast agent, is a blood pool tracer that never leaves the blood vessels and can be observed in real time and dynamically when showing microcirculation perfusion [20]. CEUS is a new technology applied in clinical practice in recent years, which can significantly improve the display rate of low-speed blood flow and evaluate the blood perfusion characteristics of organs and lesions. It is able to show the nourishing blood vessels, reflect the true characteristic blood supply, and determine the nature of tumors [21, 22].

Among the CEUS manifestations of all the 5 testicular malignant tumor cases, fast-in and fast-out enhancement was seen in 2 seminomas and 2 mixed germ cell tumors, and fast-in and slow-out enhancement was seen in 1 seminoma. Heterogeneous hyperenhancement was seen at their peak time. One testicular adenomatoid tumor presented fast-in and fast-out enhancement and slightly heterogeneous hyperenhancement at the peak time, which was similar to a testicular malignant tumor, indicating abundant blood supply inside. A testicular adenomatoid tumor is a kind of benign tumor without typical clinical manifestations. Substantially occupied lesions on gray scale ultrasound can usually be seen in the regional part of the testicle, which is with clear boundaries, homogeneous internal echo, and hypoecho or isoecho compared with the surrounding tissues [23]. Since there was only 1 patient in this group, the CEUS findings still needed to be confirmed. Two testicular hematomas did not show any enhancement on CEUS. It is not difficult to make a conclusion combined with trauma history, which provides strong evidence for the clinical diagnosis of testicular injury and the determination of injury types [24].

The reason why 1 case of testicular tuberculosis was misdiagnosed as a malignant testicular tumor in this study was that it had similar CEUS characteristics to testicular malignant tumors, which brought certain difficulties to the differential diagnosis. So, when we meet patients with diffuse nodules, details of TB history should be inquired about, because the exact clinical history data plays a suggestive role in the diagnosis of TB [25].

Ultrasonic contrast agent SonoVue is the ideal contrast agent; its characteristics are listed as follows: (1) nontoxic; (2) possible to intravenously inject; (3) circulation through the lungs, heart, and capillaries; and (4) stability of recirculation. Ultrasound contrast agents can increase the reflective difference between the tumor and normal tissue and enhance the Doppler blood flow signals inside lesions. The vascular morphology, distribution, and blood supply status of tumors can be displayed more completely. It is possible to effectively improve the detection of tumor vessels, so as to evaluate them more accurately. When coming to combined diagnosis with CDFI, CEUS is hopeful to elevate the diagnosis rate and differential diagnosis rate [26].

This study has limitations. The number of research cases is limited, and we call for further in-depth research with a larger sample size to improve the diagnostic accuracy of testicular space-occupying lesions. In future studies, I will collect more clinical samples for further verification. We will study the clinical application value of CEUS in the diagnosis, staging, and follow-up of testicular space-occupying lesions.

In conclusion, as it is noninvasive, nonradiative, and possible to observe the real-time blood perfusion of testicular occupied lesions dynamically, CEUS has a high clinical application value of the diagnosis and differential diagnosis concerning benign and malignant testicular occupied lesions. We reported for the first time the application value of CEUS as a benign and malignant diagnosis and differentiation of testicular space-occupying lesions. It has important value in the diagnosis of testicular space-occupying lesions.

## Figures and Tables

**Figure 1:** The CDFI manifestations of testicular occupied lesions: (a) abundant CDFI signals in a testicular malignant tumor; (b) absence of CDFI signals in a testicular hematoma.

**Figure 2:** The CEUS manifestations of testicular malignant tumors: (a) fast-in enhancement phase of the mass; (b) heterogeneous hyperenhancement at the peak time; (c) fast-out enhancement phase of the mass.

**Figure 3:** The CEUS manifestation of a testicular hematoma. No enhancement during the entire process ((a) 25^th^ sec, (b) 35^th^ sec, and (c) 90^th^ sec).

## Data Availability

The datasets used and/or analyzed during the current study are available from the corresponding author on reasonable request.
